The article "Segmentation and Classification of Glaucoma Using U-Net with Deep Learning Model" was published in 2022. Journal: J Healthc Eng.

# Segmentation and Classification of Glaucoma Using U-Net with Deep Learning Model

**DOI:** 10.1155/2022/1601354

**Published:** 2022-02-16

**Authors:** M. B. Sudhan, M. Sinthuja, S. Pravinth Raja, J. Amutharaj, G. Charlyn Pushpa Latha, S. Sheeba Rachel, T. Anitha, T. Rajendran, Yosef Asrat Waji

**Affiliations:** ^1^Department of Artificial Intelligence and Machine Learning, MVJ College of Engineering, Bangalore, Karnataka, India; ^2^Department of Information Science and Engineering, M. S. Ramaiah Institute of Technology, Bangalore, Karnataka, India; ^3^Department of Computer Science & Engineering, Presidency University, Bangalore, Karnataka, India; ^4^Department of Information Science and Engineering, RajaRajeswari College of Engineering, Mysore Road, Bangalore, Karnataka, India; ^5^Saveetha School of Engineering, Saveetha Institute of Medical and Technical Sciences (Deemed to be University), Chennai, Tamilnadu, India; ^6^Department of Information Technology, Sri Sairam Engineering College (Autonomous), Chennai, Tamilnadu, India; ^7^Makeit Technologies, Coimbatore, Tamilnadu, India; ^8^Department of Chemical Engineering, College of Biological and Chemical Engineering Addis Ababa Science and Technology University, Addis Ababa, Ethiopia

## Abstract

Glaucoma is the second most common cause for blindness around the world and the third most common in Europe and the USA. Around 78 million people are presently living with glaucoma (2020). It is expected that 111.8 million people will have glaucoma by the year 2040. 90% of glaucoma is undetected in developing nations. It is essential to develop a glaucoma detection system for early diagnosis. In this research, early prediction of glaucoma using deep learning technique is proposed. In this proposed deep learning model, the ORIGA dataset is used for the evaluation of glaucoma images. The U-Net architecture based on deep learning algorithm is implemented for optic cup segmentation and a pretrained transfer learning model; DenseNet-201 is used for feature extraction along with deep convolution neural network (DCNN). The DCNN approach is used for the classification, where the final results will be representing whether the glaucoma infected or not. The primary objective of this research is to detect the glaucoma using the retinal fundus images, which can be useful to determine if the patient was affected by glaucoma or not. The result of this model can be positive or negative based on the outcome detected as infected by glaucoma or not. The model is evaluated using parameters such as accuracy, precision, recall, specificity, and F-measure. Also, a comparative analysis is conducted for the validation of the model proposed. The output is compared to other current deep learning models used for CNN classification, such as VGG-19, Inception ResNet, ResNet 152v2, and DenseNet-169. The proposed model achieved 98.82% accuracy in training and 96.90% in testing. Overall, the performance of the proposed model is better in all the analysis.

The article "Segmentation and Classification of Glaucoma Using U-Net with Deep Learning Model" was published in 2022. Journal: J Healthc Eng.

## 1. Introduction

It is important to diagnose glaucoma early on, which can reduce damage and loss of vision and ensure prompt and appropriate care. The worldwide prevalence of glaucoma for people ages 40 to 80 years is 3.54%. Each one out of 200 individuals aged 40 have glaucoma, which ascends to one in eight by age 80 [1]. Various glaucoma-related risk factors have been established, where the elevated intraocular pressure (IOP) that damages the optic nerves and blood vessels is the significant one. It can lead to total damage to the optic nerves and cause vision loss, if glaucoma is left untreated. This gradual and complete damage to the optic nerves is often followed by only mild or no symptoms, so it is known as the “sneak thief of sight” [2].

Glaucoma is one of the most common causes of irreversible vision loss after cataracts worldwide, accounting for 12 percent of all blindness cases each year. The number of people affected by glaucoma between the ages of 40 and 80 is expected to rise to 111.8 million by 2040. Furthermore, 2.4 percent of all people and 4.7 percent of those aged 70 and up are at risk of developing the disorder. Glaucoma is defined as the degeneration of retinal ganglion cells (RGCs) caused by a variety of disorders. RGC degeneration may result in two major health concerns:

- Structural changes to the optic nerve head (ONH) and the nerve fiber layer
- Concurrent functional failures of the field of vision

These two glaucoma side effects might induce peripheral vision loss and, if left unchecked, blindness. Besides early detection and treatment, there is no cure for glaucoma. It is essential in developing automated techniques for detecting glaucoma early on [3]. A retinal fundus image is an essential tool for documenting the optic nerve's health, vitreous, macula, retina, and blood vessels. Ophthalmologists used a fundus camera to take the retinal image. The retinal image was used to diagnose eye disease like glaucoma. Glaucoma is a significant cause of global blindness that cannot be cured. Glaucoma disease can change the cup region's shape, which is the center portion of the ONH. The changes can be used as a parameter for the early indicator of glaucoma. The ONH transmits visual information from retina to the brain [2].  Figure 1 shows the retinal fundus images.

There are no initial glaucoma symptoms but will gradually damage the optic nerves and then results in blindness. Thus, it is crucial to detect glaucoma as early as possible so that it can prevent visual damage. Physiologically, glaucoma is indicated by increased optic cup excavation. The increasing size of the optic cup will impact the size of the optic disc, and this relation is known as a cup-to-disc ratio (CDR). It means ophthalmologists can diagnose glaucoma progression using the value of CDR measurement. The optic cup and optic disc segmentation will support to calculate the CDR from the retinal image [3]. The most noticeable symptom of glaucoma is often a loss of side vision, which might go unnoticed as the condition progresses. This is why glaucoma is sometimes referred to as the sneaky thief of vision. In the case of extreme intraocular pressure levels, headache, sudden eye pain, impaired vision, or the formation of halos around lights might occur.

- Loss of vision
- Eye redness
- Hazy eyes (specifically in infants)
- Vomiting or nausea
- Vision narrowing (tunnel vision) [4]

There are many forms of glaucoma, including angle-closure glaucoma (ACG), primary open-angle glaucoma (POAG), primary congenital glaucoma (PCG), normal-tension glaucoma (NTG), pseudoexfoliative glaucoma (XFG), traumatic glaucoma (TG), uveitic glaucoma (UG), pigmentary glaucoma (PG), and neovascular glaucoma. The forms vary between different ethnicities in intensity, complexity, and occurrence. Open-angle and angle-closure glaucoma are the two major forms of glaucoma [4].  Figure 2 is shown in optic nerve head structure.

The article "Segmentation and Classification of Glaucoma Using U-Net with Deep Learning Model" was published in 2022. Journal: J Healthc Eng.

The most common form of glaucoma is open-angle glaucoma also referred to as wide-angle glaucoma. It happens as a result of partial drainage canal blockage in which the pressure slowly rises as the fluid is not properly drained. Symptoms start from vision loss in the periphery and may not be detected until central vision is impaired. Angle-closure glaucoma caused by impulsive and aqueous drainage full blockage is often called acute glaucoma. The pressure increases exponentially, which quickly leads to vision loss. It is formed because of the angle of narrow drainage and the small and droopy iris. The iris is pulled inside the anterior angle of the eye against the trabecular mesh network (drainage canals) leading to blockage and bulging of the iris forward [5].

In most situations, this damage is caused by abnormal rise of the pressure inside the eye. The secretion rate is equalised to the drainage rate in healthy eyes. Glaucoma occurs when the drainage canal was partially or entirely blocked, leading to a surge in pressure known as intraocular pressure that affects the optic nerves used to relay signals to the brain where it is possible to perceive visual information. If this damage is left untreated, complete blindness will result. Hence, it is essential to diagnose glaucoma in early stage.

The article "Segmentation and Classification of Glaucoma Using U-Net with Deep Learning Model" was published in 2022. Journal: J Healthc Eng.

In this research, early prediction of glaucoma using deep learning technique is proposed. In this proposed deep learning model, the ORIGA dataset is used for the evaluation of glaucoma images. For segmentation, the U-Net segmentation model is implemented in this model and a pretrained transfer learning model, DenseNet-201, is used for feature extraction along with deep convolution neural network (DCNN). The DCNN approach is used for the classification, and the final results will be representing whether the glaucoma infected or not.

## 2. Related Works

Several study models have been developed by various authors for the segmentation and classification of glaucoma detection, each employing a different methodology and algorithm from the others. As will be detailed more, the majority of them are deep learning-based models with varying levels of performance analysis. The fact that retinal disease is such a terrible ailment makes it difficult to detect and distinguish between the two conditions.

The most common approach used in most of the studies to diagnose glaucoma was the acquisition of retinal scans using digital capture equipment for visual content, which was the most common procedure used in most of the studies. The scan images were then preprocessed to equalize the anomalies. During the preprocessing stage, blood vessels were segmented and depicted in order to create a vessel free image. Furthermore, feature extraction was utilized to efficiently reduce the dimensions of an image in order to represent the interesting areas of an image as a compact feature vector that could be used for precisely classifying the large amount of data collected. Techniques such as textures, pixel intensity values, FFT coefficients, and histogram models were employed in the process of feature extraction and classification. Data analysis and classification were accomplished through the use of image classification, which involved examining the numerical aspects of an image. The data set was divided into several classifications based on the results, such as normal or glaucoma, to facilitate analysis.

Prastyo et al. applied the U-Net segmentation technique to retinal fundus images in order to segment the optic cup. The segmentation of the optic cup and the optic disc aids in the achievement of improved performance in the detection of glaucoma disease. The ROI based on the optic disc image was cropped and segmented with the help of the U-Net algorithm. In order to obtain optimal training, an adaptive learning rate optimization technique was applied, and the model attained a dice coefficient rate of 98.42 percent and a loss rate of 0.15 percent during testing [6]. A model of attention-based CNN (AG-CNN) for identifying glaucoma was proposed by Li et al. and it was tested on a database known as the large-scale attention-based glaucoma database (LAG). The removal of large levels of redundancy from fundus images may result in a reduction in the accuracy and reliability of glaucoma identification. The AG-CNN model took this into consideration and made a decision on it. In this model, subnets of attention prediction, pathological region localization, and classification were combined to form an overall model. When it comes to detecting glaucoma, the model has a 96.2 percent accuracy rate and an AUC of 0.983. In several cases, the ROI was only partially highlighted, and the minor problematic regions were not correctly identified [7].

The article "Segmentation and Classification of Glaucoma Using U-Net with Deep Learning Model" was published in 2022. Journal: J Healthc Eng.

For the purpose of automatically segmenting the glaucoma images, MacCormick et al. developed a new glaucoma detection algorithm based on spatial detection. The method was developed on the basis of four assumptions: segmentation, deformation, shape, and size of the images were all taken into consideration. After a segmentation of the cup and disc of the retinal fundus images was completed, an estimation of the cup/disc ratio (CDR) in 24 cross sections was performed to generate the pCDR (CDR profile). The results were compared between healthy discs and glaucomatous discs on both external and internal validation, with the AUROC for internal validation being 99.6 percent and for external validation being 91 percent [8].

Juneja et al. proposed an artificial intelligence glaucoma expert system that was based on the segmentation of the optic cup and disc. In order to automate the identification of glaucoma, a deep learning architecture was designed, with CNN serving as the core element. In this model, two neural networks were integrated and used for segmenting images of the optic disc and cup of fundus, which were taken from different cameras. By examining 50 images, the model was able to segment the cup with 93 percent accuracy and the disc with 95.8 percent accuracy [9]. To diagnose glaucoma in retinal fundus images, Diaz-Pinto et al. used five ImageNet trained models, including the VGG-16, VGG-19, ResNet50, Inception-v3, and Xception, all of which were trained using ImageNet data. Performance study revealed that the Xception model outperformed the other models by obtaining better results, and the Xception model was then tested with five publicly accessible datasets for glaucoma diagnosis to confirm its superiority. The Xception model was more efficient than other commonly used models [10] due to its higher level of computing efficiency.

The article "Segmentation and Classification of Glaucoma Using U-Net with Deep Learning Model" was published in 2022. Journal: J Healthc Eng.

With the help of deep learning, SynaSreng et al. developed an automated two-stage model for glaucoma diagnosis and classification. Initially, the optic disc area was segmented using DeepLabv3+ architecture, but the encoder segment was replaced with several deep CNNs after the initial segmentation. For classification, a trained DCNN was employed with three approaches: transfer learning, feature descriptors learning using SVM, and constructing an ensemble of techniques in transfer learning and feature descriptors learning, respectively. It was possible to segment the optic discs using DeepLabv3+ and MobileNet architectures because of the integration of the two systems. Five separate glaucoma datasets were used in the classification process, which was done using an ensemble of algorithms. Finally, utilizing the ACRIMA dataset, DeepLabv3+ and MobileNet were able to achieve an accuracy of 99.7 percent for OD segmentation and 99.53 percent for classification using DeepLabv3+ and MobileNet [11].

To diagnose diabetic retinopathy, Mateen et al. developed a fundus image classification model that combined the VGG-19 with principal component analysis (PCA) and singular value decomposition (SVD) and used the VGG-19. The model's performance in region segmentation, feature extraction and selection, and classification has been improved by combining the Gaussian mixture model with the VGG, PCA, and SVD [12, 13]. Fu et al. employed two deep learning-based glaucoma detection techniques, multilabel segmentation network (M-Net) and disc-aware ensemble network, to detect the presence of glaucoma (DENet). Initially, M-Net was utilized to solve the segmentations of both the optic cup and the disc, and DENet was used to combine the deep hierarchical context of the global fundus image with the local optic disc region in the initial stages. The CDR was calculated based on the segmentation of the optic cup and disc in order to determine the glaucoma risk. It is possible to get accurate results from an image without segmenting it using the DENet [13].

Jiang et al. developed a new multipath recurrent U-Net model for segmenting retinal fundus image. The efficiency of the model was validated by the performance of two segmentation processes like optic cup and disc segmentation and retinal vessel segmentation. The model achieved 99.67% accuracy for optic disc segmentation, 99.50% for optic cup segmentation, and 96.42% for retinal vessel segmentation by using the Drishti-GS1 dataset [14].

Mahum et al. proposed an early-stage glaucoma diagnosis model based on deep learning-based feature extraction. Images were preprocessed in the first phase before the region of interest was retrieved using segmentation. Then, using the hybrid features descriptors, such as CNN, histogram of oriented gradients, local binary patterns, and speeded up robust features, characteristics of the optic disc were recovered from images including optic cup. Furthermore, HOG was used to extract low-level features, while the LBP and SURF descriptors were used to extract texture features. Furthermore, CNN was used to compute high-level characteristics. The feature selection and ranking technique of maximum relevance minimum redundancy was applied. Finally, multiclass classifiers such as SVM, KNN, and random forest were used to determine if fundus images were healthy or diseased [15].

The article "Segmentation and Classification of Glaucoma Using U-Net with Deep Learning Model" was published in 2022. Journal: J Healthc Eng.

Gheisari et al. proposed a new method for detecting glaucoma that combined temporal (dynamic vascular) and spatial (static structural) data. A CNN and recurrent neural network (RNN) classification model that extracts not just the spatial features in the fundus images but additionally the temporal features inherent in the consecutive images was developed. Because CNN was designed to diagnose glaucoma, it was built on spatial information encoded in images. CNN was used with RNN for increased performance in detecting glaucoma based on both temporal and spatial features [16].

## 3. Proposed Methodology

In this research, the deep learning-based models are proposed for segmentation and classification of glaucoma detection using retinal fundus images collected from ORIGA database. For segmentation, the U-Net architecture is used and a pretrained DenseNet-201 architecture was used to extract the features from the segmented image. For classification, the DCNN architecture is used to classify the images for detecting glaucoma.

### 3.1. Dataset Description

The ORIGA dataset is used in this research for evaluation [17]. The data set contains 650 images of the color retinal fundus with the extension (.jpg) and ground truth with the extension (.mat). The retinal images were collected by the Singapore Malay Eye Study (SiMES). ORIGA database shares clinical ground truth retinal images with the public and provides open access for researchers to benchmark their computer-aided segmentation algorithms. ORIGA dataset is open for online access upon request. After preprocessing, 650 image data were divided into 488 image data as training data, 162 image data as testing data [1, 6, 8, 11, and 13].

### 3.2. Segmentation Using U-Net

The deep learning algorithm-based U-Net architecture is implemented for optic cup segmentation. The U-Net architecture is the most widely used segmentation architecture for medical images. The architecture of the U-Net segmentation process is shown in Figure 3. The retinal fundus image is given as input; the ROI based on optical disc image is cropped and segmented using deep learning algorithm. The output of the segmentation will be based on the optic cup, where the optic cup outline is masked as shown in Figure 3.

The article "Segmentation and Classification of Glaucoma Using U-Net with Deep Learning Model" was published in 2022. Journal: J Healthc Eng.

Before segmenting the image, in preprocessing, the ground truth (mask) image was changed to (.png) so that an algorithm could process it. To get the Optic Disk (OD) mask, we used the equation (disc = double (mask > 0)), while for Optic Cup (OC), we employed the equation (cup = double (mask > 1)). After that, we took the region of interest (ROI) from the retinal fundus image by using the ground truth from OD to take OC's closest area.

A contracting path (left side) and an expansive path (right side) are included in this architecture, joined by multilevel skip connections (middle). Input to the contracting path is retinal fundus images, and predictions are generated from a final layer following the expansive path. Each convolution layer has filter banks, each applying 3 × 3 padded convolutions followed by a rectified linear activation unit whose functional form is *f*(*z*) = max (0, *z*) [18–20].

There are three convolutional blocks each in the contracting and expansive paths. Two convolutional layers consist of a block in the contracting path followed by a max-pooling layer with a pool size of 2 × 2. A block contains a 2 × 2 upsampling layer in the expansive path, a concatenation from the contracting path with the corresponding block (i.e., a merged layer), a dropout layer, and two convolutional layers. The connecting path includes two convolutional layers. Finally, a 1 × 1 convolutional layer with a sigmoid activation and a single filter to output pixel-wise class scores is the final output layer. Every convolution layer in blocks 1, 2, and 3 includes 112, 224, and 448 filters in the contracting path, while blocks 5, 6, and 7 include 224, 122, and 122 filters in the expansive path individually. There are 448 filters in every convolutional layer in the connecting path. The proposed DCNN differs from the original U-Net in the number of filters chosen for the model to fit into the GPU memory in each convolution layer and the use of dropouts in the expansive path.

### 3.3. DenseNet-201 with CNN

A DCNN model with pretrained DenseNet-201 is proposed in this research [21]. This DenseNet-201 model is based on deep transfer learning (DTL) as it is implemented to identify the glaucoma images from the input dataset by classifying the retinal fundus images. To extract features from the dataset, a pretrained DenseNet-201 model is used, and the DCNN model is used for classification. 256 × 256 is the input image size. The architecture of the DenseNet-201 with DCNN is shown in Figure 4.

The article "Segmentation and Classification of Glaucoma Using U-Net with Deep Learning Model" was published in 2022. Journal: J Healthc Eng.

DCNN usually performs well with a larger data set over a smaller one. TL could be useful in those CNN applications where the data set is not huge. For applications with comparatively smaller datasets, TL's concept utilizes the learned model from large datasets such as ImageNet. This removes the need for a large dataset and decreases the lengthy training time as needed when generated from scratch by the deep learning algorithm. TL is a deep learning method that uses a model trained for a single assignment as a starting point to train a model for a similar assignment. It is typically much quicker and simpler to fine-tune a TL network than training a network from scratch. By leveraging common models that have been already trained on large data sets, it allows the training of models using similar small labeled data. Training time and computing resources can be significantly decreased. With TL, the model does not need to be trained for as many epochs (a complete training period on the entire dataset) like a new model.

Because of the feature reuse possibility by various layers, the DenseNet-201 uses the condensed network that provides simple to train and highly parametrical effective models and expands variety in the following layer input and enhances the execution. On various data sets, such as CIFAR-100 and ImageNet, DenseNet-201 has shown remarkable results. Direct connections from each previous layer to every subsequent layer are added to boost connectivity in the DenseNet-201 model as shown in Figure 5.

The concatenation of feature can be mathematically expressed as

(1) $$\begin{array}{c} fc^{i}={\text{NL}}_{i}\left(fc^{0},fc^{1},\ldots ,fc^{i-1}\right). \end{array}$$

Here, NL_*i*_(∙) was a nonlinear transformation that could be described as batch normalization (BN) composite function, accompanied by a rectified linear unit function (ReLU) and a (3 × 3) convolution layer.

For ease of implementation, [*fc*^0^, *fc*^1^,…, *fc*^*i *−* *1^] indicates the feature map concatenation according to layers 0 to *i* − 1 are combined into a single tensor. Dense blocks are generated in the network architecture for downsampling purposes, divided by layers known as transition layer consisting of BN followed by a 1 × 1 convolution layer and an average 2 × 2 pooling layer. DenseNet-201's growth rate defines how dense architecture produces better results, and the “*H*” hyperparameter denotes it. Because of its structure, where feature maps were regarded as a network's global state, DenseNet-201 performs adequately well even with a minimal growth rate. Therefore, all function maps of the preceding layers have access to each successive layer. Each layer includes “*H*” feature maps to the global state where each count of input feature maps at *i*^th^ layers (*fm*)^*i*^ was expressed as

(2) $$\begin{array}{c} {\left(fm\right)}^{i}=H^{0}+H\left(i-1\right). \end{array}$$

Here, the input layer channels are given by *H*^0^. A 1 × 1 convolution layer preceding each 3 × 3 convolution layer is added to increase computational performance, which reduces the input feature maps that were usually higher than the feature maps of output H. The 1 × 1 conv layer was known as the bottleneck layer and generates feature maps. FC layers act as a classifier in the classification stage. It uses extracted features and assesses the probability of a segment in the image. The architecture of DenseNet-201 is shown in Figure 6.

The article "Segmentation and Classification of Glaucoma Using U-Net with Deep Learning Model" was published in 2022. Journal: J Healthc Eng.

To create nonlinearity and to reduce overfitting, the activation function and dropout layer are typically used. Two dense layers of 128 and 64 neurons were implemented for classification. The DenseNet-201 feature extraction model was used for binary classification preceded by the sigmoid activation function to replace the softmax activation function utilized in the DenseNet-201 design. In the FC dense layer, every neuron was FC in the prior layer. The FC layer “*i*” whose input 2D feature map was extended to a 1D feature vector can be mathematically described.

(3) $$\begin{array}{c} v^{i-1}=\text{Bernoulli}\left(p\right),\\ z^{i-1}=v^{i-1}*d^{i-1},\\ z^{i}=f\left(x^{k}z^{i-1}+u^{i}\right). \end{array}$$

Here, the Bernoulli function produces a vector *v*^*i*^*=1* randomly with a certain probability that obeys the 0-1 distribution. The dimension of the vector is *d*^*i*−1^. The dropout strategy is used by the initial two layers of the FC layer to randomly block some neurons based on a defined probability, which efficiently avoids overfitting situations in deep networks. The terms “*x*” and “*u*” describe the FC layer's respective weighting and offset parameters. The function of sigmoid activation was to convert nonnormalized outputs to 0 or 1 as binary outputs. Therefore, it helps to classify the images as nonglaucoma or glaucoma. The sigmoid function can be expressed as

(4) $$\begin{array}{c} S=\frac{1}{1+e^{-\left(\sum x_{i}\cdot z_{i}\right)}}, \end{array}$$

where the neuron output is *S*. The weights and inputs, respectively, represent *x*_*i*_ and *z*_*i*_.

## 4. Performance Analysis

The performance analysis of the proposed DCNN with the U-Net and DenseNet-201 model is assessed using the dataset in this section. The model is evaluated using parameters such as accuracy, precision, recall, specificity, and F-measure. Also, a comparative analysis is conducted for the validation of the model proposed. The output is compared to other current deep learning models used for CNN classification, such as VGG-19, Inception ResNet, ResNet 152v2, and DenseNet-169. On the MATLAB 2019a Simulink toolbox, all the experiments are implemented and carried out. The dataset is split into 75% for training and 30% for validating the performance analysis.

The article "Segmentation and Classification of Glaucoma Using U-Net with Deep Learning Model" was published in 2022. Journal: J Healthc Eng.

### 4.1. Performance Metrics

The primary objective of this research is to detect the glaucoma using the retinal fundus images, which can be useful to determine if the patient was affected by glaucoma or not. The result of this model can be positive or negative based on the outcome detected as infected by glaucoma or not. The true positive, true negative, false positive, and false negative are properly analyzed to estimate the outcome of this model.

  TP: it indicates the total predictions correctly obtained in positive cases
  FP: it indicates the total predictions incorrectly obtained in positive cases
  TN: it indicates the total predictions correctly obtained in negative cases
  FN: it indicates the total incorrect predictions in negative cases

Accuracy is the model's estimation of the performance subset. It is the primary output metric used to calculate the efficiency of the classification process. It is usually used to estimate when both the positive and negative classes are equally important. It is calculated using the following equation.

(5) $$\begin{array}{c} \text{Accuracy}=\frac{\text{TP}+\text{TN}}{\text{TP}+\text{TN}+\text{FP}+\text{FN}}\text{.} \end{array}$$

As shown in Table 1, the proposed model achieved better classification accuracy in both training and testing for classifying the glaucoma fundus images. The model obtained 98.82% training accuracy, which is 1.09% to 3.96% improved compared with other techniques. The testing accuracy is 96.90%, which is 1.36% to 5.26% increased performance than the other existing compared models. The graphical chart of the comparison is plotted in Figure 7.

Precision is a positive predictive value. It is the measure of the cumulative predictive positive value of the correctly predicted positive observation. The lower precision value reflects that a large number of false positives have affected the classification model. The measure of precision can be computed using the following equation.

(6) $$\begin{array}{c} \text{Precision}=\frac{\text{TP}}{\text{TP}+\text{FP}}. \end{array}$$

The estimation of precision is tabulated in Table 2, which shows that the proposed model has achieved better precision value than the compared models. The model obtained 98.63% precision rate in training, which was 1.1% to 4.8% improved compared with other techniques. The precision rate in testing was 96.45%, which was 1.08% to 4.9% increased performance than the other existing compared models.  Figure 8 shows the comparison of precision analysis.

The article "Segmentation and Classification of Glaucoma Using U-Net with Deep Learning Model" was published in 2022. Journal: J Healthc Eng.

The sensitivity is also referred to as recall. It is the ratio of properly predicted positive evaluation of the overall positive predictive value. The lower recall value reflects that a large number of false negative values have affected the classification model. The recall estimation can be calculated using the following equation.

(7) $$\begin{array}{c} \text{Recall}=\frac{\text{TP}}{\text{TP}+\text{FN}}. \end{array}$$

The proposed model has gained better recall or sensitivity rate as tabulated in Table 3. The model obtained 98.95% recall rate in training, which was 1.1% to 4.05% improved compared with other techniques. The recall rate in testing was 97.03%, which was 1.3% to 5.06% better performance than the other existing compared models. The comparison graph is plotted, as shown in Figure 9.

As per this model, specificity is the prediction that healthy subjects do not have the disease. It is the percentage of subjects with no illness that is tested as negative. The specificity estimation can be calculated using the following equation.

(8) $$\begin{array}{c} \text{Specificity}=\frac{\text{TN}}{\text{TN}+\text{FP}}. \end{array}$$

As shown in Table 4, the proposed model has obtained a better specificity rate than the other comparative models of deep learning.

The model obtained 98.15% specificity rate in training, which was 0.8% to 4.1% improved compared with other techniques. The specificity rate in testing was 96.33%, which was 0.6% to 6.4% better performance than the other existing compared models.  Figure 10 represents the comparison of specificity estimated.

The F-measure estimates the accuracy of the test and is defined as the weighted harmonic mean of the precision of the test and the recall. The accuracy does not take into account how the data was distributed. The F-measure is then utilized to manage the distribution problem with accuracy. When the data set has imbalance classes, it was useful. The F-measure estimation can be calculated using the following equation.

(9) $$\begin{array}{c} \text{F}-\text{measure}=\frac{2\times \text{Precision}\times \text{Recall}}{\text{Precision}+\text{Recall}}. \end{array}$$

The F-measure estimation is tabulated in Table 5, which represents that the proposed model has achieved better F-measure value than the compared models. The model obtained 98.50% F-measure rate in training, which was 0.9% to 3.7% improved compared with other techniques. The F-measure rate in testing was 96.28%, which was 0.8% to 4.7% better performance than the other existing compared models.  Figure 11 shows the comparison of F-measure analysis.

The article "Segmentation and Classification of Glaucoma Using U-Net with Deep Learning Model" was published in 2022. Journal: J Healthc Eng.

In this research, by comparing all the models like VGG-19, Inception ResNet, ResNet 152v2, and DenseNet-169, the proposed model has achieved better performance in both the training and testing stages. The least performance achieved model is Inception ResNet and DenseNet-169 has some close performance to the proposed model.

## 5. Conclusion

In this research, early prediction of glaucoma detection model using deep learning technique was proposed. In this proposed deep learning model, the ORIGA dataset was used for the evaluation of glaucoma images. 75% of the data was used for training and 25% of data was used for testing. For segmentation, the U-Net segmentation model was implemented in this model and a pretrained transfer learning model, DenseNet-201, was used for feature extraction along with DCNN. The DCNN approach was used to classify the images for glaucoma detection. The primary objective of this model was to detect the glaucoma using the retinal fundus images, which can be useful to determine whether the patient is affected by glaucoma or not. By segmenting the fundus images, the optic cup region was segmented and compared with ground truth images from the dataset. After segmentation, the features were extracted from the images using DenseNet model and classified using DCNN. The proposed model obtained 98.82% training accuracy, which was 1.09% to 3.96% higher compared with other models and the testing accuracy was 96.90%, which was 1.36% to 5.26% higher than the compared models. By analyzing the performance analysis, the results obtained by the proposed model are efficient and the reason for not achieving 100% results was due to the false positives and false negatives. In future, this imbalance issue will be sorted out by improving the classifier and reducing the threshold. This model can be useful for various medical image segmentation and classification processes like diabetic retinopathy, brain tumor detection, breast cancer detection, etc.

## Figures and Tables

**Figure 1:** Retinal fundus images: (a) healthy eye, (b) early glaucoma, (c) moderate glaucoma, and (d) deep glaucoma [2].

**Figure 2:** Structure of optic nerve head: (a) normal and (b) glaucoma [3].

**Figure 3:** U-Net architecture of segmentation [6].

**Figure 4:** U-Net output image compared with ground truth image.

**Figure 5:** Feature extraction using pretrained DenseNet-201 model and classification using DCNN [21].

The article "Segmentation and Classification of Glaucoma Using U-Net with Deep Learning Model" was published in 2022. Journal: J Healthc Eng.

**Figure 6:** DenseNet-201 architecture [21].

**Figure 7:** Graphical plot of accuracy.

**Figure 8:** Graphical plot of precision.

**Figure 9:** Graphical plot of recall.

**Figure 10:** Graphical plot of specificity.

**Figure 11:** Graphical plot of F-measure.

**Table 1:** Performance analysis of accuracy.

Models	Training	Testing
VGG-19	97.73	95.54
Inception ResNet	94.86	91.64
ResNet 152v2	97.56	93.21
DenseNet169	97.14	95.45
Proposed	98.82	96.90

**Table 2:** Performance analysis of precision.

Models	Training	Testing
VGG-19	97.30	94.70
Inception ResNet	93.81	91.52
ResNet 152v2	97.28	93.02
DenseNet169	97.49	95.37
Proposed	98.63	96.45

**Table 3:** Performance analysis of recall.

Models	Training	Testing
VGG-19	97.84	95.62
Inception ResNet	94.90	91.97
ResNet 152v2	97.62	94.05
DenseNet169	97.35	95.69
Proposed	98.95	97.03

**Table 4:** Performance analysis of specificity.

Models	Training	Testing
VGG-19	97.24	95.67
Inception ResNet	94.05	89.92
ResNet 152v2	97.28	92.73
DenseNet169	97.00	94.89
Proposed	98.15	96.33

**Table 5:** Performance analysis of F-measure.

Models	Training	Testing
VGG-19	97.52	95.39
Inception ResNet	94.79	91.55
ResNet 152v2	97.35	93.14
DenseNet169	97.07	95.09
Proposed	98.50	96.28

## Data Availability

The datasets used and/or analyzed during the current study are available from the corresponding author on reasonable request.
